# Response of Breast Cancer Cells and Cancer Stem Cells to Metformin and Hyperthermia Alone or Combined

**DOI:** 10.1371/journal.pone.0087979

**Published:** 2014-02-05

**Authors:** Hyemi Lee, Heon Joo Park, Chang-Shin Park, Eun-Taex Oh, Bo-Hwa Choi, Brent Williams, Chung K. Lee, Chang W. Song

**Affiliations:** 1 Department of Microbiology, College of Medicine, Inha University, Incheon, Korea; 2 Department of Pharmacology, College of Medicine, Inha University, Incheon, Korea; 3 Department of Therapeutic Radiology-Radiation Oncology, University of Minnesota Medical School, Minneapolis, Minnesota, United States of America; University of Pittsburgh School of Medicine, United States of America

## Abstract

Metformin, the most widely prescribed drug for treatment of type 2 diabetes, has been shown to exert significant anticancer effects. Hyperthermia has been known to kill cancer cells and enhance the efficacy of various anti-cancer drugs and radiotherapy. We investigated the combined effects of metformin and hyperthermia against MCF-7 and MDA-MB-231 human breast cancer cell, and MIA PaCa-2 human pancreatic cancer cells. Incubation of breast cancer cells with 0.5–10 mM metformin for 48 h caused significant clonogenic cell death. Culturing breast cancer cells with 30 µM metformin, clinically relevant plasma concentration of metformin, significantly reduced the survival of cancer cells. Importantly, metformin was preferentially cytotoxic to CD44^high^/CD24^low^ cells of MCF-7 cells and, CD44^high^/CD24^high^ cells of MIA PaCa-2 cells, which are known to be cancer stem cells (CSCs) of MCF-7 cells and MIA PaCa-2 cells, respectively. Heating at 42°C for 1 h was slightly toxic to both cancer cells and CSCs, and it markedly enhanced the efficacy of metformin to kill cancer cells and CSCs. Metformin has been reported to activate AMPK, thereby suppressing mTOR, which plays an important role for protein synthesis, cell cycle progression, and cell survival. For the first time, we show that hyperthermia activates AMPK and inactivates mTOR and its downstream effector S6K. Furthermore, hyperthermia potentiated the effect of metformin to activate AMPK and inactivate mTOR and S6K. Cell proliferation was markedly suppressed by metformin or combination of metformin and hyperthermia, which could be attributed to activation of AMPK leading to inactivation of mTOR. It is conclude that the effects of metformin against cancer cells including CSCs can be markedly enhanced by hyperthermia.

## Introduction

Metformin (1,1-dimethylbiguanide hydrochloride) originally derived from French lilac, is the most widely used oral hypoglycemic drug for treatment of type 2 diabetes [1], [2]. Accumulating evidences in recent years clearly showed that metformin possesses significant anti-cancer effects [2]–[9]. For instance, the incidences of various cancer and cancer-related mortality have been found to be markedly lower in type 2 diabetic patients treated with metformin than in those treated with other types of anti-diabetes drugs [7],[8]. Furthermore, metformin enhanced the response of cancers to neoadjuvant chemotherapy [9]. Numerous pre-clinical studies have shown that metformin suppresses proliferation and induces apoptotic and clonogenic death in various cancer cells [9]–[13]. Metformin has also been shown to prevent lung tumorigenesis caused by tobacco carcinogens [14] and enhance the response of experimental tumors to chemotherapy [15],[16] and radiotherapy [6]. Randomized clinical trials evaluating the anti-cancer effectiveness of metformin are in progress [2].

A number of divergent cellular and molecular mechanisms have been proposed to account for the anti-cancer effects of metformin [2]–[4],[8],[10]–[14],[17]–[20]. Metformin has been reported to disrupt oxidative phosphorylation in mitochondria, thereby decreasing ATP level and concomitantly increasing AMP level. The resultant increase in AMP/ATP ratio activates AMPK, an energy sensor, leading to inactivation of mTOR, which is known to promotes protein synthesis, cell growth, cell cycle progression and cell proliferation by activating downstream effectors signals such as S6K and 4EBP1 [21]. Therefore, the anti-cancer effect of metformin has been attributed to its ability to activate AMPK, thereby leading to down-regulation of mTOR. We have previously reported that ionizing radiation activated AMPK and that ionizing radiation and metformin synergistically activated AMPK and suppressed mTOR activity in both cultured cells in vitro and experimental tumors in vivo [6]. On the other hand, there are some indications that anti-cancer effect of metformin may be mediated by mechanisms independent of AMPK activation [2],[20].

It has become increasingly evident that small proportions of cancer cells are cancer stem cells (CSCs) (cancer stem cell-like cells or tumor initiating cells) [6],[15],[16],[22]–[25]. Such cells have been demonstrated to be resistant to conventional chemotherapy [25]–[28] or radiotherapy [6],[28]–[31], and thus frequently survive the treatments. The surviving CSCs may then cause recurrence or metastases of cancer. Importantly, metformin has been shown to preferentially kills CSCs, compared to non-CSCs, both in vitro and in vivo [2],[15],[16],[32]. Recent studies demonstrated that metformin inhibits cellular transformation and cancer stem cell growth by inhibiting the associated inflammatory response [33] or by decreasing expression of CSC-specific gene [34]. We have also reported that metformin preferentially kills CSCs, compared to non-CSCs, and increases the radiosensitivity of CSCs, and enhances the response of experimental tumors to radiotherapy [6].

It is well-established that moderate hyperthermia at 39–43°C kills cancer cells and sensitizes cancer cells to chemotherapy or radiotherapy [35]–[38]. Interestingly, human breast CSCs have been reported to be resistant than non-CSCs to hyperthermia applied with water-bath whereas CSCs and non-CSCs were equally vulnerable to nanoparticle-mediated photothermal therapy [39]. A recent study reported that human breast CSCs were resistant to radiotherapy, but hyperthermia with optically activated gold nanoshells markedly increased the sensitivity of CSCs to radiotherapy [40],[41]. In the present study, we show that metformin is preferentially cytotoxic to CSCs relative to non-CSCs and that hyperthermia markedly increases the metformin cytotoxicity against CSCs. For the first time, we observed that hyperthermia activates AMPK, thereby suppressing mTOR. Such an activation of AMPK by hyperthermia appeared to play an important role in the hyperthermia-induced potentiation of metformin cytotoxicity against cancer cells, particularly against CSCs.

## Materials and Methods

### Cell lines

MCF-7 (p53 wild-type) and MDA-MB-231 (p53 mutated) human breast cancer cells and MIA PaCa-2 human pancreatic cancer cells were obtained from the American Type Culture Collection (ATCC) (Manassas, VA).

### Clonogenic cell survival

Cells were plated into T25 plastic tissue culture flasks with 4 ml RPMI 1640 medium (GIBCO Invitrogen, Grand Island, NY) containing 10% (v/v) bovine fetal calf serum (FCS), penicillin (50 units/ml), and streptomycin (50 µg/ml). The cells were incubated overnight under standard tissue culture conditions (i.e., under a humidified 5% CO_2_ atmosphere at 37°C), and used for following experiments. *Effect of metformin alone*: Cells were incubated with 0.5–10 mM metformin for 48 h, gently rinsed twice with PBS, and cultured in regular medium under standard culture conditions for 18 days. The colonies formed were fixed, stained with crystal violet, the numbers of colonies containing more than 50 cells were counted, and clonogenic survival was calculated [6],[38]. *Effect of heating:* Culture flasks with cells were tightly closed, the neck area of flasks was wrapped with wax paper, and the flasks were immersed into a preheated water bath at 42°C [38]. After heating for 1 h at 42°C, cells were cultured under standard culture conditions and clonogenic survival was assessed. *Effect of combination of hyperthermia and metformin*: Cells were heated with 5 mM metformin at 42°C for 1 h, and then incubated at 37°C for 47 h. After removing metformin and rinsing twice with PBS, cells were cultured in regular medium under standard culture conditions, and clonogenic survival was assessed. *Effect of low doses of metformin*. The plasma concentration of metformin in type 2 diabetes patient treated with metformin is constantly elevated to 6–30 µM. To mimic such a clinical situation, we cultured breast cancer cells in mediate containing 30 µM metformin for 18 days and determined the clonogenic survival. Fever-range whole-body hyperthermia in combination with chemotherapy is one of the cancer therapy modalities [37]. We therefore investigate the combined effect of fever-range hyperthermia with 30 µM metformin by heating the cells at 39.5°C for 6 h and culturing the cells for 18 day with 30 µM metformin at 37°C.

### Cell proliferation and cell cycle distribution

*Changes in cell numbers:* Into T25 plastic tissue culture flasks, about 6×10^4^ cells were plated, incubated overnight at 37°C, and then incubated with regular medium with 5 mM metformin. After incubation for varying lengths of time, cells were trypsinized and cells that excluded trypan blue were counted using a hemocytometer. The effect of hyperthermia on cell proliferation was studied by heating the cells in regular medium at 42°C for 1 h and then incubating at 37°C. The effect of a combination of metformin and hyperthermia on cell proliferation was studied by heating the cells at 42°C for 1 h with metformin and then incubating at 37°C with metformin. *Immunofluorescence microscopy for PCNA:* Cell proliferation was also assessed by immunohistological examination of PCNA (proliferating cell nuclear antigen) expression. Cells treated with metformin alone, heating alone or combined as described above, were fixed with 4% (v/v) paraformaldehyde at −20°C for 20 min, washed three times with PBS, and permeabilized with 0.2% (v/v) Triton X-100/PBS for 10 min. After treating with blocking buffer (3% [w/v] BSA/PBS) for 30 min at room temperature, cells were incubated overnight at 4°C with mouse monoclonal antibody directed against PCNA (Santa Cruz Biotechnology, Santa Cruz, CA) diluted 1∶100 in 1% (w/v) BSA/PBS. After washing three times with PBS, the cells were incubated with FITC-conjugated secondary antibody (1∶500) (Molecular Probes, Eugene, OR) for 1 h at room temperature. Cells were mounted on microscopy glass slides with mounting medium containing DAPI, and cell proliferation was assessed by measuring the fluorescence intensity of PCNA and DAPI with fluorescence microscopy. *Cell cycle distribution.* Cells were treated with metformin and heating alone or in combination as described above for cell proliferation experiment. The cells were then labeled with propidium iodide and the cell cycle distribution was assessed using flow cytometry.

### Determination of CSCs of MCF-7 and MIA PaCa-2 cells

The CSCs of MCF-7 cells are known to express CD44^high^/CD24^low^ [6],[15],[16],[25],[30],[32]. The proportions of MCF-7 cells expressing CD44^high^/CD24^low^ before and after treatment with metformin alone, heating alone, or combined were determined. The CD44^high^/CD24^low^ cells were identified by the method we previously described [6]. Briefly, after treating the cells in culture flasks with metformin and heating alone or combined, cells were dispersed into single cells by trypsin treatment, washed, and suspended in PBS. Cells were next incubated for 20 min with FITC-conjugated anti-CD44 antibody (BD Biosciences, Franklin Lakes, NJ) followed by incubation with phycoerythrine-conjugated anti-CD24 antibody (BioLegend, San Diego, CA) for 20 min in the dark at 4°C. After washing with PBS containing 1% (v/v) FCS, CD44^high^/CD24^low^ cells were identified with flow cytometry [6],[15],[27]–[29],[32], and the % of CD44^high^/CD24^low^ cells was estimated. The same method was applied to identify CD44^high^/CD24^high^ cells, which are CSCs of MIA PaCa-2 cells [25].

### Sphere Formation

CSCs are known to grow as spheres when cultured in suspension, and thus sphere formation has been used to identify CSCs [6]. MCF-7 cells were plated in special culture plates (ultralow attachment plate) (1000 cells/plate) in serum free RPMI medium supplemented with 20 ng/ml BGF, 20 ng/ml EGF, 5 µg/ml bovine insulin and 2% (v/v) B27. Metformin was added to the media (0.5–5 mM), the plates were sealed with wax-paper and then immersed into water-bath at 42°C for 1 h. Thereafter, the cells were incubated for 8 days under the standard culture conditions. The numbers of spheres with diameter >50 µm were counted under a microscope [6].

### Western blotting

After various treatments, i.e. metformin and heating alone or combined, cells were dissolved in lysis buffer containing protease inhibitors on ice for 30 min. The lysates were resolved by SDS-polyacrylamide gel electrophoresis (PAGE) and transferred to nitrocellulose membranes. After blocking with 1% (w/v) nonfat dry milk in Tris-buffered saline with 0.05% (v/v) Tween 20, the membranes were incubated with primary antibody followed by a goat anti-rabbit or anti-mouse IgG conjugated with horseradish peroxidase, and the immunoreactive bands were visualized with chemiluminescence (SUPEX, NeuroNex, Korea). (All antibodies were obtained from Cell Signaling Technology, Beverly, MA).

### Small interfering RNA transfection

siRNA duplex targeting human AMPKα (5′-CCAUACCCUUGAUGAAUUA-3) was purchased from Dharmacon (Lafayette, CO). Transfection of cells with the siRNA duplexes at 50 nM final concentrations was performed using LipofectAMINE 2000 (Invitrogen). AccuTarget™ siRNA (Invitrogen, Carlsbad, CA) was used as a negative control.

### Statistics

Statistical significance of variances between group means was analyzed using either Student *t* test or ANOVA. Differences with p<0.05 were considered to be statistically significant.

## Results

### AMPK/mTOR pathway

Figure 1 shows the effects of heating alone and metformin alone or in combination on the AMPK/mTOR signaling pathway. In MCF-7 cells, heating at 42°C for 1 h and subsequent incubation at 37°C for 47 h caused a gradual activation of AMPK, as shown by an increase in the extent of phosphorylation of the protein, over the 48 h incubation. Heating also significantly increased the phosphorylation of ACC, a known target of AMPK, but suppressed the phosphorylation of mTOR and its downstream effector S6K. Figure 1B shows that a 48 h incubation with 5 mM metformin at 37°C increased the levels of p-AMPK and p-ACC and suppressed the expression of p-mTOR and p-S6K. Heating the cells at 42°C for 1 h with 5 mM metformin followed by incubation at 37°C markedly upregulated p-AMPK and downregulated p-mTOR and p-S6K. The effects of heating alone, metformin alone or the combination on the activation of AMPK/mTOR signaling pathway in MDA-MB-231 cells (Figs. 1C and D) were essentially identical to those in MCF-7 cells. The effects of heating at temperatures lower than 42°C alone or in combination with 5 mM metformin on the expression of AMPK/mTOR pathways are shown in Figure 1E. Heating at 39.5–41°C for 1 h upregulated p-AMPK and downregulated p-mTOR in temperature dependent manner. Combinations of heating at 39.5–41°C and 5 mM metformin were significantly more effective than heating or metformin alone to activate AMPK/mTOR pathway. Incubation of MCF-7 cells for 6 h with 30 µM metformin alone at 37°C or heating at 39.5°C for 6 h activated AMPK/mTOR pathway and combination of 30 µM metformin treatment with 39.5°C heating markedly upregulated AMPK/mTOR pathway (Fig. 1F).

**Figure 1:** Western blotting of AMPK/mTOR pathway in MCF-7 and MDA-MB-231 cells treated with hyperthermia and metformin. (A, C) Cells were heated at 42°C for 1 h and then incubated at 37°C for 47 h (total 48 h treatment). (B, D) The effects of metformin alone were studied by incubating cells with 5 mM metformin for 48 h at 37°C. The combined effects of metformin and heating were studied by heating the cells at 42°C for 1 h with 5 mM metformin and then incubating at 37°C for 47 h. (E) The combined effects of metformin and heating were studied by heating the cells at 39.5–41°C for 1 h with 5 mM metformin and then incubating at 37°C for 47 h. (F) The combined effects of metformin and heating were studied by heating the cells at 39.5°C for 6 h with 30 µM metformin and then incubating at 37°C for 47 h. Experiments were repeated 4–5 times and the representative results are shown.

### Clonogenic death of cancer cells

Figures 2A and C show the clonogenically surviving cell fraction of MCF-7 cells and MDA-MD-231 cells, respectively, after a 48 h of incubation at 37°C with 0.5–10 mM metformin alone, or metformin in combination with a 1 h heating at 42°C. The clonogenic survival declined sharply as the metformin concentration was increased up to 5 mM in both cell lines. The incubation with 5 mM metformin at 37°C decreased the survival of MCF-7 and MDA-MB-231 cells to about 60% (Fig. 2A) and 20% (Fig. 2C) of control values, respectively. The p53 in MDA-MB-231cells is mutated, which may be the reason why MDA-MB-231 cells are more sensitive than MCF-7 cells to metformin [42].Treatment with 10 mM metformin was only slightly more effective than that with 5 mM to reduce clonogenic survival in both cell lines. Heating at 42°C for 1 h without metformin reduced clonogenic survival by 20% in MCF-7 cells and 35% in MDA-MB-231 cells, and heating potentiated the effect of metformin at all the metformin concentrations tested, i.e. 0.5–10 mM, in both cell lines (Figs. 2A and C). We then investigated whether the cell deaths caused by metformin alone or in combination with hyperthermia are related to the AMPK activity by transfecting the cells with AMPK siRNA. The insets in Figures 2B and D show that AMPK was almost completely blocked by AMPK siRNA transfection in both cell lines. As shown in Figures 2B and D, the clonogenic deaths caused by metformin alone or in combination with heating were markedly reduced by AMPK siRNA transfection. To clearly assess the role of AMPK in combined effect on cell survival, the survival curves for the combination of heating with metformin were normalized for the cell death caused by heating alone in Figures 2B and C. It can have seen that AMPK played a critical role in clonogenic cell death caused by metformin alone or in combination with heating. As shown in Figure 2E, continuous exposure of MCF-7 cells to 30 µM metformin for 18 days reduced cell survival to 78.4% and heating at 39.5°C for 6 h reduced the survival to 80.5%. Cell survival decreased to 54.1% when cells were heated at 39.5°C for 6 h and cultured for 18 days with 30 µM metformin. The combined effect of fever-range hyperthermia for 6 h and continued exposure to metformin on cell survival was merely additive.

**Figure 2:** Clonogenic surviving fraction of MCF-7 and MDA-MB-231 cells after treated with hyperthermia and metformin. (A, C) Cells were incubated with 0–10 mM of metformin for 48 h at 37°C, or cells were heated at 42°C for 1 h with 0–10 mM metformin or without metformin and then incubated for 47 h at 37°C. After the 48 h metformin treatments, cells were washed and cultured for 18 days in regular media and the colonies formed were counted. Means of 6 experiments ±1 S.E. are shown. The decrease in cell survival by heating alone was statistically significant, and the survival of cells treated with the combination of heating and metformin was statistically smaller than that by metformin alone at all the metformin concentrations tested. (B, D) To elucidate the role of AMPK in the cell death caused by metformin alone or in combination with heating, cells were transfected with AMPK siRNA or control siRNA. The insets are Western blots for AMPK after transfection with control siRNA or AMPK siRNA. The transfected cells were treated with metfomin alone, heat alone or in combination with heating as described above and their clonogenic survival was determined. Cell death caused by the combined treatment was normalized for the death caused by heating alone. Means of 5 experiments ±1 S.E. are shown. The decreases in the effect of metformin by siRNA transfection were statistically significant both at 37°C and 42°C. (E) MCF-7 cells in medium containing 30 µM metformin were heated at 39.5°C for 6 h and then cultured at 37°C for 18 days. The effects of heating alone, metformin alone and combined on % survival of cells are shown. Means of 7 experiments ±1 S.E. are shown. The survival of cells treated with metformin in combination with heating was statistically smaller than that caused by metformin alone and heating alone.

### Cell proliferation

Incubation with 5 mM metformin markedly suppressed the proliferation of MCF-7 cells (Fig. 3A). Heating for 1 h at 42°C alone slightly suppressed cell proliferation, but heating significantly enhanced the effect of metformin to suppress cell proliferation. The differences among the results of 4 different treatment groups at 72 h were statistically significant (p<0.05). As shown in Figures 3B and C, transfection of MCF-7 cells with AMPK siRNA reduced the effects of metformin alone or with heating to suppress cell proliferation. The immunohistological staining for PCNA expression in MCF-7 (Fig. 4A) and the ratio of the fluorescence intensity of PCNA to that of DAPI (Fig. 4B) also demonstrated that cell proliferation was suppressed markedly by metformin and slightly by heating, and to a greater extent by combination of metformin and heating. Silencing AMPK with siRNA suppressed markedly the effects of metformin and only slightly the effect of heating to reduce PCNA expression. Silencing the AMPK activity significantly reduced the effect of combination of heating and metfomin to inhibit PCNA expression.

**Figure 3:** Proliferation of MCF-7 human breast cancer cells treated with hyperthermia and metformin. Numbers of viable cells (trypan blue excluding cells) were counted with a hemocytometer after incubations for 0–72 h. (A) 37°C; incubated in regular medium. 37°C + Met; incubated in medium containing 5 mM metformin. 42°C; heated at 42°C for 1 h in regular medium and incubated. 42°C + Met; heated at 42°C for 1 h and incubated in medium containing 5 mM metformin. The variances in cell numbers among the 4 groups at 72 h were statistically significant (ANOVA). The cell number of 42°C + Met group was statistically smaller than that of 37°C + Met group by student t-test. (B, C) MCF-7 cells were transfected with control siRNA or AMPK siRNA and the effects of metformin and heating or combined on cell proliferation were studied. Effect of siRNA to suppress the effect of metformin alone or in combination with heating was statistically significant.

**Figure 4:** Cell proliferation was studied with immunostaining for PCNA and DAPI in MCF-7 cells. (A) Cells transfected with AMPK siRNA or control siRNA were incubated for 48 h at 37°C with or without 5 mM metformin. The effect of heating at 42°C for the first 1 h of 48 h incubation with or without 5 mM metformin was also studied. Following treatments, cells were immunostained for PCNA and DAPI, and the immunofluorescence intensity of PCNA and DAPI was determined with immunofluorescence microscopy. (B) Ratio of PCNA/DAPI fluorescence intensity observed in A. Means of 5 experiments ±1 S.E. is shown. The decrease in PCNA/DAPI fluorescence intensity by metformin was statistically significant at both 37°C and 42°C, and siRNA transfection significantly reduced the effect of metformin to decrease the PCNA/DAPI fluorescence intensity.

### Cyclins and Cell Cycle Distribution

As shown in Figure 5, in MCF-7 cells, heating at 42°C for 1 h caused little changes in the levels of cyclin A, cyclin B1, cyclin D1 and cyclin E whereas an incubation with 5 mM metformin for 72 h caused a gradual reduction in the level of cyclin D1 but not in other cyclins. The combination of heating and metformin treatment decreased the levels of all the cyclins. Figure 5B shows that, in both MCF-7 cells and MDA-MB-231 cells, expression of cyclin D1 was almost completely suppressed by the combination of heating and metformin in control cells, but such inhibition of cyclin D1 was markedly suppressed by silencing AMPK with siRNA. These results demonstrated that AMPK plays an important role in the cyclin D1 expression. The change in cell cycle distribution of MCF-7 cells is shown Figure 5C. Heating at 42°C for 1 h followed by 47 h incubation at 37°C exerted little effect on cell cycle distribution. Incubation with 5 mM metformin for 48 h caused a small increase in G2/M cell population and slight decreases in S cell and G1 cell populations. Although these changes in cell cycle distribution by metformin treatment were small, the changes were statistically significant (p<0.05). The population of apoptotic cells slightly increased by metformin alone. The 9.8% of cells were apoptotic cell after combined treatment of heating and metformin as compared to 3.6% prior to treatment. This increase in apoptosis was statistically significant (p<0.05) albeit the increase was small.

**Figure 5:** Western blotting of cyclins expression in MCF-7 and MDA-MB-231 cells treated with hyperthermia and metformin. (A) 42°C; Cells were heated at 42°C for 1 h and then incubated at 37°C for 24–72 h. Met; Cells were incubated with or without 5 mM metformin for 24–72 h at 37°C. 42°C + Met; Cells were heated at 42°C for 1 h with or without 5 mM metformin and then incubated at 37°C for 24–72 h. (B) Cells were transfected with AMPK siRNA or control siRNA, and incubated with or without 5 mM metformin for 72 h at 37°C. Effects of 1 h heating at 42°C at the inception for 72 h treatment with or without 5 mM metformin were also studied. Representative results out of several repeated studies are shown. (C) Changes in cell cycle distribution after 42°C heating for 1 h followed by 47 h incubation at 37°C, 48 h treatment with 5 mM metformin at 37°C, or combination of heating and metformin. The increase in G2/M cells, decreased in S cells and increase in apoptotic cells by metformin treatment was statistically significant. The increase in apoptotic cell population in the Heat + Met group as compared with that in Met group was statistically significant.

### Cancer Stem cells

**CD44^high^/CD24^low^ and CD44^high^/CD24^high^ cells:** Figure 6A shows the flow cytometry analysis of the effects of metformin and heating alone or combined on the proportions of CD44^high^/CD24^low^ cells, i.e. CSCs, of MCF-7 cells. In a representative study shown in Figure 6A, incubation of MCF-7 cells with different concentrations of metformin decreased CD44^high^/CD24^low^ cell population in dose dependent manner: 5 mM metformin for 48 h at 37°C decreased the proportion of CD44^high^/CD24^low^ cells from control value of 2.78% to 1.29%. Such decline in the proportions of CD44^high^/CD24^low^ cells indicated that metformin preferentially eliminated CSCs in comparison with non-CSCs. Heating of MCF-7 cells at 42°C for 1 h caused small reduction in the proportion of CD44^high^/CD24^low^ cells, and heating the cells at 42°C for the first 1 h of 48 h treatment with 1 mM or 5 mM metformin reduced the proportions of CD44^high^/CD24^low^ cells to 0.51% and 0.08%, respectively. The results of 4 replicate experiments are summarized in Figure 6B. The reductions of CSCs by combination of heating and metformin were significantly greater than the reductions by either of them alone. It is clear that heating at 42°C for 1 h potentiated the efficacy of metformin to selectively kill CSCs in MCF-7 cells. Figure 6C is the representative result of flow cytometry analysis for the effects of heating and metformin alone or combined on the proportion of CD44^high^/CD24^high^ cells, CSCs of MIA PaCa-2 cells. About 6.55% of MIA PaCa-2 cells were CD44^high^/CD24^high^ cells before treatment, and an incubation of the MIA PaCa-2 with 1 mM metformin for 48 h at 37°C decreased the proportion of CD44^high^/CD24^high^ cell to 4.53%. Heating MIA PaCa-2 cells at 42.5°C for 1 h slightly reduced the proportion of CD44^high^/CD24^high^ cells to 5.33%, but heating the cells with 1 mM metformin at 42.5°C reduced the proportion of CD44^high^/CD24^high^ cells to 2.48%.

**Figure 6:** Percent of CSCs in MCF-7 human breast cancer cells treated with hyperthermia and metformin. (A) Cells were incubated with 0–5 mM metformin for 48 h at 37°C, dispersed to single cells and analyzed for CD44^high^/CD24^low^ cells (CSCs) with FACS. The effect of heating alone was studied by heating the cells at 42°C for 1 h followed by 47 h incubation at 37°C. The combined effect of heating and metformin was studied by heating the cells for 1 h at 42°C with metformin and then incubating at 37°C for 47 h. (B) Experiments described in A were repeated four times and the average of % of CSCs was obtained. Averages of 5 experiments ±1 S.E. are shown. The decreases in CSCs by 1 mM and 5 mM alone were statistically significant. The decrease in CSCs by heating at 42°C for 1 h was also statistically significant. The combinations of heating and metformin were statistically more effective than metformin alone. (C) MIA PaCa-2 cells were incubated with 0–10 mM metformin for 48 h at 37°C, dispersed to single cells and analyzed for CD44^high^/CD24^high^ cells (CSCs) with FACS. The effect of heating alone was studied by heating the cells at 42.5°C for 1 h followed by 47 h incubation at 37°C. The combined effect of heating and metformin was studied by heating the cells for 1 h at 42.5°C with metformin and then incubating at 37°C for 47 h. (D, E) MCF-7 cells were plated in ultralow attachment plate (1,000 cells/plate) in sphere media. Metformin was added to the media (0.5–5 mM), then heating at 42°C for 1 h. Thereafter, the cells were incubated for 8 days under the standard culture conditions. The numbers of spheres with diameter >50 µm were counted under a microscope. The combinations of heating and metformin were statistically more effective than metformin alone.

**Sphere Formation:** When 1,000 MCF-7 cells were plated and cultured in ultra-attachment culture plates for 8 days, about 24 spheres were formed, as shown in Figures 6D and E. The number of sphere formed decreased to 16 when 1,000 MCF-7 cells were cultured with 1 mM metformin. This decrease was statistically significant (p<0.05). Heating at 42°C for 1 h and subsequent incubation for 8 days at 37°C slightly reduced sphere formation, but heating significantly enhanced to the effect of metformin to inhibit sphere formation. For example, only 12 spheres were formed when cells were treated with heating in combination with 1 mM metformin.

## Discussion

In the present study, metformin was cytotoxic to MCF-7 and MDA-MB-231 human breast cancer cells and MIA PaCa-2 human pancreatic cancer cells, preferentially to cancer stem cells. Heating at 42°C for 1 h was slightly cytotoxic to cancer cells and cancer stem cells, but it markedly enhanced the cytotoxicity of metformin against cancer cells, preferentially cancer stem cells. The heat-induced enhancement of metformin cytotoxicity appeared to be mediated by potentiation of AMPK activation.

The PTEN/PI3K/Akt/mTOR signaling pathway plays a crucial role in protein synthesis, cell cycle progression, cell proliferation, and cell survival [2]–[4],[21],[43]–[45]. It has been known that this pathway is frequently mutated and dysregulated in malignant cells, particularly in CSCs [43]–[45]. Apart from Akt, AMPK is a major regulator of mTOR. Whereas Akt upregulates mTOR, AMPK downregulates mTOR. AMPK, a master regulator of cellular energy homeostasis, is activated by an upstream kinase LKB1, a tumor suppressor protein, in response to various cellular stresses. Metformin disrupts mitochondrial respiration, thereby increasing the AMP/ATP ratio leading to activation of AMPK [2]–[4],[10]–[14],[46]. As shown in Figure 1, incubation of MCF-7 and MDA-MB-231 cells with 5 mM metformin for 48 h at 37°C significantly increased phosphorylation (activation) of AMPK and reduced expression of p-mTOR. Figure 2 shows that silencing AMPK with siRNA reduced the extent of metformin-induced clonogenic cell death, showing that AMPK/mTOR pathway plays an important role in the metformin-induced cell death.

Heating at 42°C for 1 h also increased the level of p-AMPK and reduced that of p-mTOR (Fig. 1). To the best of our knowledge, our study is the first to show that hyperthermia activates AMPK, and thereby suppresses mTOR activity. The mechanism underlying the activation of AMPK by heating is unclear, but it would be reasonable to suggest that heating interferes with cellular respiration and thus reduces ATP supply, thereby increasing AMP/ATP ratio leading to AMPK activation. Importantly, the combination of heating and metformin was highly effective to elevate p-AMPK level and to reduce the levels of p-mTOR and its downstream effector p-S6K (Fig. 1). Such effect on AMPK/mTOR pathway may account for the enhancement of metformin-induced clonogenic cell death by heating (Fig. 2). In support of this conclusion, inhibition of AMPK with siRNA significantly reduced the combined effects of heating and metformin to cause clonogenic cell death (Fig. 2). In this context, we [6] and others [47],[48] reported that irradiation activated AMPK and that irradiation increased the metformin-mediated activation of AMPK.

Metformin suppressed the proliferation of MCF-7 cells as determined both by cell counting (Fig. 3) and PCNA expression (Fig. 4). Heating alone slightly reduced cell proliferation but it markedly enhanced the metformin-induced suppression of cell proliferation (Figs. 3 and 4). Inhibition of AMPK with siRNA alleviated the suppression of cell proliferation caused by metformin, alone or in combination with heating (Figs. 3 and 4). These results show that metformin-induced suppression of cell proliferation is dependent on AMPK activity. We investigated whether the suppression of cell proliferation caused by metformin alone or in combination with heating was associated with changes in cyclin activity. In MCF-7 cells, heating alone caused little change in cyclin D1 levels whereas metformin alone caused considerable suppression in the cyclin D1 level (Fig. 5A). Interestingly, whereas only cyclin D1 was suppressed by the treatment with metformin alone, all cyclin B1, cyclin D1, and cyclin E levels were suppressed when cells were treated with a combination of metformin and heating. The metformin-induced reduction in cyclin D1 level that we observed in the present study is consistent with reports by others that metformin suppresses the levels of cyclin D1 and causes cell cycle arrest at the G1 checkpoint [4],[11],[13],[49]. Inhibition of AMPK activity in MCF-7 cells by siRNA prohibited the decline in cyclin D1 level caused by the combination of metformin and heating (Fig. 5B). These results clearly demonstrated that AMPK is an important player in the suppression of cyclin D1 level and cell proliferation by metformin alone or in combination with heating. The decline in cyclin D1 by metformin, particularly in combination with heating, may have suppressed the progression of G1 cells to S phase, as indicated by the reduction of S phase cell population (Fig. 5C). Metformin treatment also caused G2/M arrest. These perturbations of cell cycle progression together with apoptosis may account for the retardation of cell proliferation by metformin alone or in combination with heating (Fig. 3).

Emerging evidence indicates that small proportions of cancer cells are cancer stem cells (CSCs) and that all CSCs must be eradicated for complete control of cancer [6],[15],[16],[22]–[25]. Incubation of MCF-7 cells with metformin for 48 h at 37°C reduced the proportion of CD44^high^/CD24^low^ cells, known to be the CSCs of breast cancer, in a dose-dependent manner (Fig. 6). Likewise, metformin also reduced the proportion of CD44^high^/CD24^high^, CSCs of MIA PaCa-2 pancreatic cancer cells. These results clearly indicated that metformin is preferentially cytotoxic to cancer stem cells, relative to non-cancer stem cells, which is in good agreement with recent reports by us as well as others [2],[6],[15],[16],[32]. Figure 6 also show that the proportion of CSCs among slightly decreased by heating at 42°C for 1 h. Such a decline in the proportion of CSCs implies that CSCs may be more vulnerable than non-CSCs to heating. This is a significant finding since CSCs has been known to be more resistant than non-CSCs to radiation [6],[28]–[31] and chemotherapy drugs [24]–[28]. On the contrarily to our results, other investigators recently report that CSCs were resistant to water bath heating as compared with non-CSCs [39]. However, these investigators observed that CSCs could be killed by photothermal therapy using multiwalled carbon nanotubes [39]. Importantly, we found that that hyperthermia potentiated the efficacy of metformin to selectively eliminate CSCs (Figs. 6A and C). It remains unclear why CSCs are more susceptible than are non-CSCs to metformin alone or in combination with heating. In view of the increasing evidence that the PI3K/Akt/mTOR survival pathway is activated to a much greater extent in CSCs compared to non-CSCs and [43]–[45], it is highly possible that inactivation of mTOR by metformin alone or in combination with hyperthermia is more damaging to CSCs than to non-CSCs. Hyperthermia has been known to sensitize cancer cells to radiotherapy or chemotherapy [35]–[38]. Hyperthermia using optically activated gold nanoshells has recently been demonstrated to sensitize breast CSCs to radiotherapy through suppressing the intrinsic capacity of CSCs to repair radiation-induced DNA damage [40],[41]. It is of note that, as our present study shows, hyperthermia increases the sensitivity of CSCs to metformin, and we have previously reported that metformin increased the radiosensitivity of CSCs in vitro and markedly increased the response of tumors to radiation [6]. These observations strongly indicate that combination of hyperthermia, radiation and metformin may be a potentially effective trimodality anti-cancer treatment.

One may ask whether the metformin doses used in our in vitro experiments are relevant to clinical application of metformin for cancer treatment. The plasma metformin concentration of type 2 diabetes patients treated with metformin is constantly elevated to 6–30 µM range [13],[18]. Moreover, the metformin concentrations in tissues of diabetic mice have been reported to be several-fold higher than that in circulating blood [50]. The results shown in Figure 2E and our previous observation [6] indicated that continuous exposure to 30 µM metformin kills considerable proportions of cancer cells, and that mild heating at 39.5°C (fever range temperature) for 6 h significantly enhances the effect of 30 µM metformin against cancer cells. In this respect, as shown in Figure 1F, AMPK/mTOR pathway in MCF-7 cells was activated by 6 h incubation with 30 µM metformin at 37°C or 6 h heating at 39.5°C, and the pathway was further activated by the combination of 30 µM metformin treatment with 39.5°C heating.

## Conclusions

Metformin killed cancer cells and suppressed the proliferation of cancer cells by downregulating cyclin D1. Hyperthermia alone at 42°C for 1 h was slightly cytotoxic and it markedly potentiated the cytotoxicity of metformin against cancer cells. Importantly, the cytotoxicity of metformin alone or in combination with hyperthermia was significantly greater to CSCs than that to non-CSCs. The major molecular target of metformin alone or in combination with hyperthermia appeared to be AMPK/mTOR pathway. Combination of metformin and hyperthermia was highly effective to activate AMPK. Given that metformin is the drug most widely used by type 2 diabetes patients, and that the drug is relatively safe and inexpensive, combination of metformin and hyperthermia is a potentially useful adjuvant treatment to radiotherapy or chemotherapy for cancer.

## References

[1] WittersLA (2001) The blooming of the French lilac. J Clin Invest 108: 1105–1107.1160261610.1172/JCI14178PMC209536

[2] RattanR, Ali FehmiR, MunkarahA (2012) Metformin: an emerging new therapeutic option for targeting cancer stem cells and metastasis. J Oncol 2012: 928127.2270148310.1155/2012/928127PMC3373168

[3] KourelisTV, SiegelRD (2012) Metformin and cancer: new applications for an old drug. Med Oncol 29: 1314–1327.2130199810.1007/s12032-011-9846-7

[4] Ben SahraI, Le Marchand-BrustelY, TantiJF, BostF (2010) Metformin in cancer therapy: a new perspective for an old antidiabetic drug? Mol Cancer Ther 9: 1092–1099.2044230910.1158/1535-7163.MCT-09-1186

[5] Gonzalez-AnguloAM, Meric-BernstamF (2010) Metformin: a therapeutic opportunity in breast cancer. Clin Cancer Res 16: 1695–1700.2021555910.1158/1078-0432.CCR-09-1805PMC2840206

[6] SongCW, LeeH, DingsRP, WilliamsB, PowersJ, et al (2012) Metformin kills and radiosensitizes cancer cells and preferentially kills cancer stem cells. Sci Rep 2: 362.2250021110.1038/srep00362PMC3324825

[7] EvansJM, DonnellyLA, Emslie-SmithAM, AlessiDR, MorrisAD (2005) Metformin and reduced risk of cancer in diabetic patients. BMJ 330: 1304–1305.1584920610.1136/bmj.38415.708634.F7PMC558205

[8] LiD, YeungSC, HassanMM, KonoplevaM, AbbruzzeseJL (2009) Antidiabetic therapies affect risk of pancreatic cancer. Gastroenterology 137: 482–488.1937542510.1053/j.gastro.2009.04.013PMC2735093

[9] JiralerspongS, PallaSL, GiordanoSH, Meric-BernstamF, LiedtkeC, et al (2009) Metformin and pathologic complete responses to neoadjuvant chemotherapy in diabetic patients with breast cancer. J Clin Oncol 27: 3297–3302.1948737610.1200/JCO.2009.19.6410PMC2736070

[10] DowlingRJ, ZakikhaniM, FantusIG, PollakM, SonenbergN (2007) Metformin inhibits mammalian target of rapamycin-dependent translation initiation in breast cancer cells. Cancer Res 67: 10804–10812.1800682510.1158/0008-5472.CAN-07-2310

[11] AlimovaIN, LiuB, FanZ, EdgertonSM, DillonT, et al (2009) Metformin inhibits breast cancer cell growth, colony formation and induces cell cycle arrest in vitro. Cell Cycle 8: 909–915.1922149810.4161/cc.8.6.7933

[12] LiuB, FanZ, EdgertonSM, DengXS, AlimovaIN, et al (2009) Metformin induces unique biological and molecular responses in triple negative breast cancer cells. Cell Cycle 8: 2031–2040.1944003810.4161/cc.8.13.8814

[13] ZakikhaniM, DowlingRJ, SonenbergN, PollakMN (2008) The effects of adiponectin and metformin on prostate and colon neoplasia involve activation of AMP-activated protein kinase. Cancer Prev Res (Phila) 1: 369–375.1913898110.1158/1940-6207.CAPR-08-0081

[14] MemmottRM, MercadoJR, MaierCR, KawabataS, FoxSD, et al (2010) Metformin prevents tobacco carcinogen—induced lung tumorigenesis. Cancer Prev Res (Phila) 3: 1066–1076.2081067210.1158/1940-6207.CAPR-10-0055PMC3192328

[15] HirschHA, IliopoulosD, TsichlisPN, StruhlK (2009) Metformin selectively targets cancer stem cells, and acts together with chemotherapy to block tumor growth and prolong remission. Cancer Res 69: 7507–7511.1975208510.1158/0008-5472.CAN-09-2994PMC2756324

[16] IliopoulosD, HirschHA, StruhlK (2011) Metformin decreases the dose of chemotherapy for prolonging tumor remission in mouse xenografts involving multiple cancer cell types. Cancer Res 71: 3196–3201.2141516310.1158/0008-5472.CAN-10-3471PMC3085572

[17] ZakikhaniM, DowlingR, FantusIG, SonenbergN, PollakM (2006) Metformin is an AMP kinase-dependent growth inhibitor for breast cancer cells. Cancer Res 66: 10269–10273.1706255810.1158/0008-5472.CAN-06-1500

[18] Martin-CastilloB, Vazquez-MartinA, Oliveras-FerrarosC, MenendezJA (2010) Metformin and cancer: doses, mechanisms and the dandelion and hormetic phenomena. Cell Cycle 9: 1057–1064.2030537710.4161/cc.9.6.10994

[19] TomimotoA, EndoH, SugiyamaM, FujisawaT, HosonoK, et al (2008) Metformin suppresses intestinal polyp growth in ApcMin/+ mice. Cancer Sci 99: 2136–2141.1880363810.1111/j.1349-7006.2008.00933.xPMC11159964

[20] RattanR, GiriS, HartmannLC, ShridharV (2011) Metformin attenuates ovarian cancer cell growth in an AMP-kinase dispensable manner. J Cell Mol Med 15: 166–178.1987442510.1111/j.1582-4934.2009.00954.xPMC3822503

[21] SchmelzleT, HallMN (2000) TOR, a central controller of cell growth. Cell 103: 253–262.1105789810.1016/s0092-8674(00)00117-3

[22] Al-HajjM, WichaMS, Benito-HernandezA, MorrisonSJ, ClarkeMF (2003) Prospective identification of tumorigenic breast cancer cells. Proc Natl Acad Sci U S A 100: 3983–3988.1262921810.1073/pnas.0530291100PMC153034

[23] LoboNA, ShimonoY, QianD, ClarkeMF (2007) The biology of cancer stem cells. Annu Rev Cell Dev Biol 23: 675–699.1764541310.1146/annurev.cellbio.22.010305.104154

[24] O'BrienCA, KresoA, JamiesonCH (2010) Cancer stem cells and self-renewal. Clin Cancer Res 16: 3113–3120.2053070110.1158/1078-0432.CCR-09-2824

[25] BaoQ, ZhaoY, RennerA, NiessH, SeeligerH, et al (2010) Cancer stem cells in pancreatic cancer. Cancers 2: 1629–1641.2428117810.3390/cancers2031629PMC3837327

[26] LouH, DeanM (2007) Targeted therapy for cancer stem cells: the patched pathway and ABC transporters. Oncogene 2: 1357–1360.10.1038/sj.onc.121020017322922

[27] ZhouBB, ZhangH, DamelinM, GelesKG, GrindleyJC, et al (2009) Tumour-initiating cells: challenges and opportunities for anticancer drug discovery. Nat Rev Drug Discov 8: 806–823.1979444410.1038/nrd2137

[28] FrosinaG (2009) DNA repair and resistance of gliomas to chemotherapy and radiotherapy. Mol Cancer Res 7: 989–999.1960900210.1158/1541-7786.MCR-09-0030

[29] BaoS, WuQ, McLendonRE, HaoY, ShiQ, et al (2006) Glioma stem cells promote radioresistance by preferential activation of the DNA damage response. Nature 444: 756–760.1705115610.1038/nature05236

[30] PhillipsTM, McBrideWH, PajonkF (2006) The response of CD24(-/low)/CD44+ breast cancer-initiating cells to radiation. J Natl Cancer Inst 98: 1777–1785.1717947910.1093/jnci/djj495

[31] BaumannM, KrauseM, HillR (2008) Exploring the role of cancer stem cells in radioresistance. Nat Rev Cancer 8: 545–554.1851193710.1038/nrc2419

[32] Vazquez-MartinA, Oliveras-FerrarosC, Del BarcoS, Martin-CastilloB, MenendezJA (2011) The anti-diabetic drug metformin suppresses self-renewal and proliferation of trastuzumab-resistant tumor-initiating breast cancer stem cells. Breast Cancer Res Treat 126: 355–364.2045853110.1007/s10549-010-0924-x

[33] HirschHA, IliopoulosD, StruhlK (2013) Metformin inhibits the inflammatory response associated with cellular transformation and cancer stem cell growth. Proc Natl Acad Sci U S A 110: 972–977.2327756310.1073/pnas.1221055110PMC3549132

[34] BaoB, WangZ, AliS, AhmadA, AzmiAS, et al (2012) Metformin inhibits cell proliferation, migration and invasion by attenuating CSC function mediated by deregulating miRNAs in pancreatic cancer cells. Cancer Prev Res (Phila) 5: 355–364.2208668110.1158/1940-6207.CAPR-11-0299PMC3786260

[35] SugaharaT, van der ZeeJ, KampingaHH, VujaskovicZ, KondoM, et al (2008) Kadota Fund International Forum 2004. Application of thermal stress for the improvement of health, 15-18 June 2004, Awaji Yumebutai International Conference Center, Awaji Island, Hyogo, Japan. Final report. Int J Hyperthermia 24: 123–140.1828358910.1080/02656730701883675PMC2765467

[36] DewhirstMW, VujaskovicZ, JonesE, ThrallD (2005) Re-setting the biologic rationale for thermal therapy. Int J Hyperthermia 21: 779–790.1633886110.1080/02656730500271668

[37] BullJM, ScottGL, StrebelFR, NagleVL, OliverD, et al (2008) Fever-range whole-body thermal therapy combined with cisplatin, gemcitabine, and daily interferon-α: A description of a phase I-II protocol. Int J Hyperthermia 24: 649–662.1860859410.1080/02656730802104740

[38] ParkHJ, ChoiEK, ChoiJ, AhnKJ, KimEJ, et al (2005) Heat-induced up-regulation of NAD(P)H:quinone oxidoreductase potentiates anticancer effects of beta-lapachone. Clin Cancer Res 11: 8866–8871.1636157610.1158/1078-0432.CCR-05-0818

[39] BurkeAR, SinghRN, CarrollDL, WoodJCS, D'AgostinoRB, et al (2012) The resistance of breast cancer stem cells to conventional hyperthermia and their sensitivity to nonoparticle-mediated photothermal therapy. Biomaterials 33: 2961–2970.2224555710.1016/j.biomaterials.2011.12.052PMC3286596

[40] AtkinsonRL, ZhangM, DiagaradjaneP, PeddibhotlaS, ContrerasA, et al (2010) Thermal enhancement with optically activated gold nanoshells sensitizes breast cancer stem cells to radiation therapy. Sci Transl Med 2: 55ra79.10.1126/scitranslmed.3001447PMC412331320980696

[41] PelicciPG, DaltonP, OrecchiaR (2011) Heating cancer stem cells to reduce tumor relapse. Breast Cancer Res 13: 305.2157527810.1186/bcr2847PMC3218927

[42] BuzzaiM, JonesRG, AmaravadiRK, LumJJ, DeBerardinisRJ, et al (2007) Systemic treatment with the antidiabetic drug metformin selectively impairs p53-deficient tumor cell growth. Cancer Res 67: 6745–6752.1763888510.1158/0008-5472.CAN-06-4447

[43] ZhouJ, WulfkuhleJ, ZhangH, GuP, YangY, et al (2007) Activation of the PTEN/mTOR/STAT3 pathway in breast cancer stem-like cells is required for viability and maintenance. Proc Natl Acad Sci U S A 104: 16158–16163.1791126710.1073/pnas.0702596104PMC2042178

[44] EylerCE, FooWC, LaFiuraKM, McLendonRE, HjelmelandAB, et al (2008) Brain cancer stem cells display preferential sensitivity to Akt inhibition. Stem Cells 26: 3027–3036.1880203810.1634/stemcells.2007-1073PMC2739007

[45] HillR, WuH (2009) PTEN, stem cells, and cancer stem cells. J Biol Chem 284: 11755–11759.1911794810.1074/jbc.R800071200PMC2673242

[46] RochaGZ, DiasMM, RopelleER, Osório-CostaF, RossatoFA, et al (2011) Metformin amplifies chemotherapy-induced AMPK activation and antitumoral growth. Clin Cancer Res 17: 3993–4005.2154351710.1158/1078-0432.CCR-10-2243

[47] SanliT, RashidA, LiuC, HardingS, BristowRG, et al (2010) Ionizing radiation activates AMP-activated kinase (AMPK): a target for radiosensitization of human cancer cells. Int J Radiat Oncol Biol Phys 78: 221–229.2061562510.1016/j.ijrobp.2010.03.005

[48] ZannellaVE, CojocariD, HilgendorfS, VellankiRN, ChungS, et al (2011) AMPK regulates metabolism and survival in response to ionizing radiation. Radiother Oncol 99: 293–299.2171503710.1016/j.radonc.2011.05.049

[49] Ben SahraI, LaurentK, LoubatA, Giorgetti-PeraldiS, ColosettiP, et al (2008) The antidiabetic drug metformin exerts an antitumoral effect in vitro and in vivo through a decrease of cyclin D1 level. Oncogene 27: 3576–3586.1821274210.1038/sj.onc.1211024

[50] WilcockC, BaileyCJ (1994) Accumulation of metformin by tissues of the normal and diabetic mouse. Xenobiotica 24: 49–57.816582110.3109/00498259409043220

